The article "Fibronectin enhances tumor metastasis through B7‐H3 in clear cell renal cell carcinoma" was retracted in 2025. Reasons: duplicated images; unreliable data; unreliable results or conclusions.

# Fibronectin enhances tumor metastasis through B7‐H3 in clear cell renal cell carcinoma

**DOI:** 10.1002/2211-5463.13280

**Published:** 2021-10-03

**Authors:** Jinjing Xie, Meiyun Sun, Dongze Zhang, Chunyang Chen, Simin Lin, Guangbo Zhang

**Affiliations:** ^1^ Medical College of Soochow University Suzhou China; ^2^ Jiangsu Institute of Clinical Immunology The First Affiliated Hospital of Soochow University Suzhou China

**Keywords:** B7‐H3, fibronectin, clear cell renal cell carcinoma, tumor metastasis

## Abstract

B7 homolog 3 (B7‐H3) plays an important role in tumor biology, but the molecular mechanism underlying the role of B7‐H3 in tumor metastasis remains unclear. In this article, our analysis of The Cancer Genome Atlas database suggested that B7‐H3 expression is associated with poor prognosis of patients with clear cell renal cell carcinoma (ccRCC). B7‐H3 knockdown affected the expression of metastasis‐related genes and significantly suppressed the metastasis of ccRCC cells, but it had no significant effect on the proliferation of ccRCC cells. Database analysis revealed a strong positive correlation between B7‐H3 and fibronectin (FN) in ccRCC cells, and further study also confirmed that FN interacts with B7‐H3. Silencing FN expression inhibited the migration and invasion of ccRCC cells, whereas exogenous FN promoted the migration and invasion of ccRCC cells, which was accompanied by activation of kinases [namely, phosphorylated (p)‐phosphoinositide 3‐kinase, p‐protein kinase B, p‐p38 and p‐extracellular regulated protein kinase]. B7‐H3 knockdown abolished the prometastatic effect of FN. In conclusion, our data suggest that B7‐H3 binds to exogenous FN and promotes the metastasis of ccRCC cells.

## Graphical abstract

In this study, we explored the clinical significance and prognostic relationship of B7 homolog 3 (B7‐H3) in clear cell renal cell carcinoma (ccRCC). We report the novel discovery that B7‐H3 interacts with plasma fibronectin in promoting ccRCC metastasis. Cotargeting fibronectin and B7‐H3 may have potential as a new therapeutic intervention strategy for ccRCC treatment.

**Abbreviations**
AKT: protein kinase B
B7‐H3: B7 homolog 3
ccRCC: clear cell renal cell carcinoma
co‐IP: coimmunoprecipitation
EMT: epithelial–mesenchymal cell transformation
ERK: extracellular regulated protein kinase
FN: fibronectin
KO: knockout
mAb: monoclonal antibody
MAPK: mitogen‐activated protein kinase
MMP9: matrix metallopeptidase 9
NC: negative control
p‐: phosphorylated
PI3K: phosphoinositide 3‐kinase
RCC: renal cell carcinoma
RT‐qPCR: real‐time quantitative PCR
shRNA: short hairpin RNA

As a malignant epithelial cell tumor with clear cytoplasm, clear cell renal cell carcinoma (ccRCC) is one of the most common renal malignancies in adults [1], consisting of 80% of all cases of renal cell carcinoma (RCC) [2]. Symptoms of metastatic spread are often detected at the diagnosis of ccRCC. Currently, surgical resection, targeted drug therapy and antibody‐based immunotherapy are the primary treatment options [3], but challenges in treatment still exist. About 30% of patients after surgical treatment will experience cancer recurrence, and the 5‐year survival rate of patients is less than 10% [4]. In fact, tumor invasion and metastasis is the main reason for RCC tumor treatment failure and death of patients [5]. Therefore, it is necessary to explore the mechanism underlying RCC metastasis.

The article "Fibronectin enhances tumor metastasis through B7‐H3 in clear cell renal cell carcinoma" was retracted in 2025. Reasons: duplicated images; unreliable data; unreliable results or conclusions.

B7 homolog 3 (B7‐H3) is a member of the B7 family that acts as a second signal to regulate the initiation of T cell immune response. Although early reports showed that B7‐H3 plays a costimulatory role in immune regulation and promotes the activation and proliferation of T cells through CD28 signaling [6, 7], subsequent studies also demonstrated that tumor‐expressing B7‐H3 functions as a cosuppressive molecule to inhibit T cell immune response, promote tumor proliferation and promote aggressiveness [8]. For example, high expression of B7‐H3 in non‐small cell lung cancer leads to their escape from antitumor immunity [9]. B7‐H3 combined with PD‐1 antibody therapy can improve patient survival [10, 11]. B7‐H3 plays an inhibitory role in T cell immune response, mostly because of the effect of multiple cytokines on the tumor microenvironment [12]. B7‐H3 also plays an important role in tumor progression [13]. B7‐H3 is expressed at a low level in normal tissues and blood vessels [14], but its expression is abnormally up‐regulated in prostate cancer, oral cancer, colorectal cancer and osteosarcoma and is positively correlated with poor prognosis [15, 16, 17, 18]. This strongly suggested that B7‐H3 may be a promising target for the development of therapeutic agents in destroying metastatic tumor cells. In addition, the tumor‐promoting effects of B7‐H3 include promoting tumor angiogenesis, improving the sensitivity of tumor cells to drug therapy and radiotherapy, enhancing cell invasion and metastasis, and affecting cell metabolism [19]. Previous studies have shown that B7‐H3 is abnormally high expressed in ccRCC tissues and vasculature [20, 21], and this is related to its poor prognosis [22, 23]. However, the metastasis mechanism of B7‐H3 remains largely unclear.

Fibronectin (FN), a high‐molecular‐weight glycoprotein component of the extracellular matrix, contains three forms, namely, cellular FN, plasma FN and fetal FN, which all contain several ligand binding domains [24, 25]. FN mediates a series of signal transduction activation pathways, thereby regulating cellular processes, such as adhesion, migration, proliferation and differentiation [26, 27]. Cancer metastasis is initiated from the separation of metastatic cells from primary tumor through blood/lymphatic vessels to different locations, followed by depositing and growing in adjacent locations [28]. Epithelial–mesenchymal cell transformation (EMT), which is regarded as a hallmark behavior of cells in tumor metastasis, is mainly manifested as loss of polarity and adhesion of cells and the ability to invade and metastasize [29, 30].

The article "Fibronectin enhances tumor metastasis through B7‐H3 in clear cell renal cell carcinoma" was retracted in 2025. Reasons: duplicated images; unreliable data; unreliable results or conclusions.

In this study, we reported that elevated B7‐H3 expression in ccRCC is associated with the metastasis and poor prognosis, and we provided the evidence that FN can form a complex with B7‐H3 to activate several kinase pathways and promote the EMT and invasion of ccRCC.

## Materials and methods

### The Cancer Genome Atlas data

The ccRCC data were downloaded from Gene Expression Profiling Interactive Analysis [The Cancer Genome Atlas (TCGA), Provisional]. We analyzed all aspects of samples with reliable data. Log rank test was performed to determine disease‐free survival. Pearson correlation coefficient between B7‐H3 and FN was calculated.

### Major reagents

Fetal bovine serum (04‐001‐1ACS; Biological Industries, Shanghai, China), lentiviral (GenePharma, China), SYBR Green Master Mix (Q121–02‐AA; Vazyme), Lipofectamine 3000 (L3000015; Invitrogen, CA, USA), RNA‐Quick Purification Kit (RN001; Yishan Biotechnology), PrimeScript™ RT Master Mix kit (RR036A; Takara), PE anti‐B7‐H3 Ig (331606; BioLegend, CA, USA), FITC anti‐B7‐H3 Ig (FAB1027F; R&D), B7‐H3 mouse monoclonal antibody (mAb; 66481‐1‐Ig; Proteintech), FN mouse mAb (66042‐1‐Ig; Proteintech, CA, USA), E‐cadherin mouse mAb (14472; Cell Signaling Technology, Boston, MA, USA), N‐cadherin Rabbit mAb (13116; Cell Signaling Technology), matrix metallopeptidase 9 (MMP9) Rabbit mAb (ab76003; Abcam, Milton, Cambridge, UK), phosphoinositide 3‐kinase (PI3K; 4249; Cell Signaling Technology), phosphorylated (p)‐PI3K (17366; Cell Signaling Technology), protein kinase B (AKT; 4691; Cell Signaling Technology), p‐AKT (4060, Cell Signaling Technology), extracellular regulated protein kinase (ERK; 4695; Cell Signaling Technology), p‐ERK (4370; Cell Signaling Technology), p38 (8690; Cell Signaling Technology), p‐p38 (4511; Cell Signaling Technology), protein A + G agarose (P2055; Beyotime), B7‐H3 Ig (14058; Cell Signaling, USA) were used in this study.

### Cell lentivirus transfection and small interfering RNA transfection

The human ccRCC cell lines 786‐O and ACHN were purchased from the Cell Bank of the Chinese Academy of Sciences, cultured in DMEM with 10% fetal bovine serum and 1% penicillin and streptomycin, and placed in an incubator at 37 °C and 5% CO_2_. Transfection of B7‐H3 short hairpin RNA (shRNA) and negative control (NC) shRNA was performed with a lentiviral expression vector (MOI (Multiplicity of infection): 20). A total of 4 μg·mL^−1^ puromycin was used to screen positive cells. Human FN small interfering RNA (5′–3′: GAUCCUGUCUACUUCACAATT) and NC small interfering RNA were transfected with Lipofectamine 3000 as a carrier. After 48 h, cell efficiency of interference was confirmed by Western blot. Follow‐up experiments were carried out.

The article "Fibronectin enhances tumor metastasis through B7‐H3 in clear cell renal cell carcinoma" was retracted in 2025. Reasons: duplicated images; unreliable data; unreliable results or conclusions.

### Total RNA extraction and RT‐qPCR

RNA‐Quick Purification Kit and PrimeScript™ RT Master Mix kit were used in total RNA extraction and cDNA synthesis, respectively. AceQ qPCR SYBR Green Master Mix (without ROX) kit was used to perform real‐time quantitative PCR (RT‐qPCR). The specific scheme was conducted in accordance with the instructions of the reagent manufacturer. All primers used in this experiment are listed in Table S1.

### Flow cytometry

The 786‐O and ACHN cells in the exponential growth phase were detached from the culture flasks and centrifuged, diluted to a cell density of 1 × 10^6^ cells·mL^−1^, and 50 μL of cell suspension was added into each flow tube, followed by the addition of 1 μL flow antibody. After incubating the cells at 4 °C in the dark for 30 min (min), they were washed and detected by the flow cytometry.

### Western blotting

The cells were lysed with radioimmunoprecipitation assay cell lysis buffer for 5 min and then sonicated, and the protein concentration was measured. Total protein (20 μg) was separated by 10% SDS/PAGE and then transferred to poly(vinylidene difluoride) membrane, blocked with 5% skimmed milk, followed by incubation with primary antibodies, such as mAbs anti‐B7‐H3 Ig, anti‐FN Ig, anti‐E‐cadherin Ig, anti‐N‐cadherin Ig, anti‐MMP9 Ig, anti‐PI3K Ig, anti‐p‐PI3K Ig, anti‐AKT Ig, anti‐p‐AKT Ig, anti‐ERK Ig and anti‐p‐ERK Ig overnight at 4 °C. The membrane was then incubated with the secondary antibody at room temperature for 1 h, added with a chemiluminescent solution after washing. A Chemi Doc^TM^ MP Imaging System was used for detection.

### Cell migration and invasion experiments

In the migration assay, 786‐O and ACHN cells were digested and centrifuged and then resuspended in serum‐free medium. A total of 200 μL of cell suspension was taken and inoculated into an 8‐μm Transwell chamber with 3 × 10^4^ cells·well^−1^. In the invasion assay, Matrigel was added to the Transwell chamber 2 h in advance and then added with the cell suspension. After 24 h, the chamber was removed for crystal violet staining. Under a microscope, five fields of view were randomly taken from each well for photographing, and the average number of cells passing through the chamber was calculated.

The article "Fibronectin enhances tumor metastasis through B7‐H3 in clear cell renal cell carcinoma" was retracted in 2025. Reasons: duplicated images; unreliable data; unreliable results or conclusions.

### *In* *vivo* mouse experiments

Animal experiments were conducted under the approval of the Institutional Animal Care and Use Committee of Soochow University (Suzhou, China). Five‐week‐old SPF Balb/c male mice (Shanghai Laboratory Animal Research Center, Shanghai, China) were randomly divided into two groups (LV (Lentivirus‐normal control)‐NC group and LV‐B7‐H3 group), with seven mice in each group. The mice were subcutaneously injected with ACHN‐LV‐NC (ACHN is a clear cell renal carcinoma cell line) and ACHN‐LV‐B7‐H3 cell lines at the same side. At day 60, all mice were sacrificed by neck dislocation, and the tumors were taken for immunohistochemistry experiments.

### Coimmunoprecipitation

The cells were lysed with immunoprecipitation lysis buffer, added with goat anti‐mouse IgG and protein A + G agarose, and shaken at 4 °C for 1 h. Supernatant was collected by centrifugation, then added with 1 μg anti‐B7‐H3 mAb and shaken overnight at 4 °C. After adding protein A + G agarose and 3 h of shaking, the cells were washed and centrifuged with PBS to collect the protein. After performing metal mixing bath at 95 °C for 5 min, western blotting was then conducted.

### Immunochemistry

The mouse tissues were dehydrated in the tissue fixative, embedded into paraffin, and sliced. After melting the wax and dehydration, the tissues were added with anti‐B7‐H3 mAb overnight at 4 °C and incubated with the secondary antibody at 37 °C for 1 h. Then the tissues were washed with PBST and stained with hematoxylin. The scoring standard of immunohistochemistry was based on four levels.

### Data analysis

The Student’s *t*‐test was used to compare the two groups, and the ANOVA was used to compare multiple groups. The correlation was analyzed by Pearson’s correlation coefficient. The statistical difference was expressed as follows: *P < 0.05; **P < 0.01; ***P < 0.001.

## Results

### High expression of B7‐H3 was associated with poor prognosis of ccRCC

The B7‐H3 molecule has been shown to be abnormally expressed in several types of tumor tissues and is considered as one of the potential indicators of tumor treatment and prognosis. To understand the role of B7‐H3 and FN in ccRCC, we first comprehensively analyzed its expression using the Gene Expression Profiling Interactive Analysis database and found that the mRNA levels of B7‐H3 and FN were higher on ccRCC (Fig. 1A,C). More importantly, Kaplan–Meier survival analysis showed that patients with ccRCC with high‐expressed B7‐H3 molecules often showed a shorter disease‐free survival when compared with those with low‐expressed B7‐H3 (Fig. 1B), but the expression of FN 1 had no significant effect on the disease‐free survival of patients with ccRCC (Fig. 1D). These findings demonstrated that a high expression of B7‐H3 in ccRCC was correlated with a poor prognosis of patients with ccRCC.

The article "Fibronectin enhances tumor metastasis through B7‐H3 in clear cell renal cell carcinoma" was retracted in 2025. Reasons: duplicated images; unreliable data; unreliable results or conclusions.

**Fig. 1:** Analysis of B7‐H3 mRNA expression in tumors and its clinical prognosis from TCGA database. (A) B7‐H3 mRNA expression levels in resected ccRCC tissues and adjacent noncancerous tissue. (B) Kaplan–Meier analysis of disease‐free survival as a function of high or low expression of B7‐H3. (C) FN 1 mRNA expression levels in resected ccRCC tissues and adjacent noncancerous tissue. (D) Kaplan–Meier analysis of disease‐free survival as a function of high or low expression of FN 1. *P < 0.05. TPM, Transcripts Per Kilobase of exon model per Million mapped reads.

### The effect of B7‐H3 on the migration, invasion and proliferation of ccRCC cells

To further study the effect of B7‐H3 molecules on the biological functions of ccRCC cells, we knocked down B7‐H3 expression from human RCC 786‐O and ACHN cell lines using shRNA. The silencing efficiency of B7‐H3 in these knockout (KO) cell lines was determined through examining their mRNA and protein levels (Fig. S1, Fig. 2A,B). We speculated that silence of B7‐H3 may affect tumor migration and invasion. As expected, the Transwell experiment showed that the migration and invasion of the B7‐H3‐KO 786‐O cells was significantly down‐regulated when compared with the control 786‐O cells (Fig. 2C). Similar findings were observed in B7‐H3‐KO ACHN cells (Fig. 2D). Thus, B7‐H3 expression was found to promote the migration and invasion of ccRCC cells.

**Fig. 2:** Construction of B7‐H3‐KO 786‐O and ACHN cell lines. (A, B) Western blotting was used to detect the knockdown efficiencies of B7‐H3 protein expression in 786‐O and ACHN cell lines. (C, D) Transwell experiment to detect the cell migration and invasion capabilities of the control and B7‐H3‐KO ccRCC cells. Values are expressed as means ± SD (*t*‐tests, *n* = 3). **P < 0.01, ***P < 0.001, B7‐H3 control group vs. B7‐H3‐KO group; 25 μm (C, D).

### Changes in the expression of metastasis‐related genes in ccRCC cells after knocking down the expression of B7‐H3

We next examined whether knockdown of B7‐H3 could affect the expression of metastasis‐related genes in the 786‐O and ACHN cell lines. Here, the results showed that the mRNA levels of N‐cadherin, MMP9, Integrin α5 and Integrin β1 in B7‐H3‐KO cells were significantly down‐regulated when compared with control cells. However, E‐cadherin expression was up‐regulated (Fig. 3A,B). It is speculated that B7‐H3 can regulate the invasion and metastasis of ccRCC cells through changes of the composition of the extracellular matrix.

The article "Fibronectin enhances tumor metastasis through B7‐H3 in clear cell renal cell carcinoma" was retracted in 2025. Reasons: duplicated images; unreliable data; unreliable results or conclusions.

**Fig. 3:** Changes in genes related to cell migration and invasion after knocking down the expression of B7‐H3. (A, B) RT‐qPCR detects the expression of E‐cadherin, N‐cadherin, MMP9, Integrin α5 and Integrin β1 genes in the B7‐H3‐KO and control 786‐O and ACHN cells assayed by RT‐qPCR. Values are expressed as means ± SD (*t*‐tests, *n* = 3). *P < 0.05, **P < 0.01, ***P < 0.001, B7‐H3 control group vs. B7‐H3‐KO group.

### B7‐H3 interacted with FN

FN is one of the main components of the extracellular matrix. We performed gene expression correlation analysis using the TCGA database and found that the mRNA expression of B7‐H3 and FN was positively correlated in ccRCC (Fig. 4A). Our previous study observed that ELISA boards coated with FN polyclonal antibody (AF1918; R&D Systems) can also identify B7‐H3 molecules (data not shown), indicating that B7‐H3 and FN may form a natural complex. Subsequently, co‐IP experiments confirmed the interaction of B7‐H3 and FN in both 786‐O and ACHN cells (Fig. 4B,C). More interestingly, the expression of FN protein was significantly down‐regulated in B7‐H3‐KO cells compared with control cells (Fig. 4D,E). For further confirmation, we subcutaneously injected the B7‐H3‐KO ACHN cells and control cells into immunodeficient mice to establish a nude mouse model, and FN expression was determined after 6 weeks. Similar down‐regulation of FN was detected in B7‐H3‐KO ACHN cells (Fig. 4F). These data therefore confirmed the interaction of B7‐H3 and FN in ccRCC cells.

**Fig. 4:** B7‐H3 interacts with FN. (A) TCGA database analysis of B7‐H3 and the correlation coefficient of FN’s two genes. (B, C), The interaction of B7‐H3 with FN in 786‐O and ACHN cells detected by co‐IP assay. (D, E) The expression of FN in the B7‐H3‐KO and control 786‐O and ACHN cells assayed by western blotting. (F) The expression of FN in the B7‐H3‐KO and control ACHN cells isolated from immunodeficient mice as assayed by immunohistochemical staining. After 6 weeks of injection, tumor tissues were collected and immunohistochemical methods were used to detect FN expression levels in tumor tissues. Values are expressed as means ± SD (*t*‐tests, *n* = 3). *P < 0.05, **P < 0.01 B7‐H3, control group vs. B7‐H3‐KO group. Scale bars: 25 μm (F).

### FN promoted cell migration and invasion partially through B7‐H3

We next investigated the role that FN plays in ccRCC metastasis. The protein level of FN was knocked down from 786‐O and ACHN cells by small interfering RNA (Fig. S2). Cell migration and invasion in the si‐FN group were found to be significantly reduced compared with the si‐control group, indicating that FN promoted cell migration and invasion (Fig. 5A,B). The same result was also reported in the study of Ou *et al*. [31]. To examine whether FN was important for B7‐H3‐mediated cell migration, we incubated exogenous FN with 786‐O and ACHN cells. The results showed up‐regulated FN level in these cells as examined by western blotting (Fig. 5C,D), suggesting that exogenous FN can be deposited on the cells. More interestingly, the deposition of FN on the cells was significantly reduced on B7‐H3‐KO cells (Fig. 5C,D). Further Transwell experiments showed that the exogenous FN could enhance migration and invasion of the control 786‐O and ACHN cells, but not B7‐H3‐KO cells (Fig. 5E,F). These data suggested that FN promotes migration and invasion of ccRCC cells dependent in part on B7‐H3.

The article "Fibronectin enhances tumor metastasis through B7‐H3 in clear cell renal cell carcinoma" was retracted in 2025. Reasons: duplicated images; unreliable data; unreliable results or conclusions.

**Fig. 5:** FN binds to B7‐H3 and promotes cell migration and invasion. (A, B) Migration and invasion ability of si‐NC and si‐FN groups examined by transwell assay. (C, D) The binding level of exogenous FN to the control and B7‐H3‐KO cells. (E, F) Migration and invasion ability of the control and B7‐H3‐KO cells that were cultured with exogenous FN. Values are expressed as means ± SD (*t*‐tests, *n* = 3). Values are expressed as means ± SD (*t*‐tests, *n* = 3). *P < 0.05, **P < 0.01, ***P < 0.001, FN control group vs. si‐FN group (A, B); *P < 0.05, **P < 0.01, ***P < 0.001, B7‐H3 control vs. FN‐treated control and KO cells. Scale bars: 25 μm (A, B, E, F).

### Exogenous FN activated PI3K/AKT and p38/ERK mitogen‐activated protein kinase signaling pathway dependent on B7‐H3

To further explore the molecular mechanism of metastasis, we first examined the expression of metastasis‐related genes. It was observed that exogenous FN could significantly promote the expression of E‐cadherin and inhibit the expression of MMP9 and N‐cadherin in the control 786‐O and ACHN cells, but not in B7‐H3‐KO cells (Fig. 6A,B). Furthermore, exogenous FN could noticeably up‐regulate the phosphorylation levels of PI3K, AKT, p38 and ERK in the control 786‐O and ACHN cells (Fig. 6C,D). However, such effect was not observed in the B7‐H3‐KO cells after adding with exogenous FN. These data indicated that exogenous FN might promote EMT process of ccRCC cells through activating the PI3K/AKT and p38/ERK mitogen‐activated protein kinase (MAPK) signaling pathways dependent on B7‐H3.

**Fig. 6:** Activation of PI3K/AKT and p38/ERK MAPK signaling by FN. (A, B) The expression of EMT‐related proteins in FN‐treated control and KO cells. (C, D) The expression of signaling pathway‐related proteins in FN‐treated control and KO cells. Values are expressed as means ± SD (*t*‐tests, *n* = 3). *P < 0.05, **P < 0.01, ***P < 0.001, B7‐H3 control vs. FN‐treated control and KO cells.

The article "Fibronectin enhances tumor metastasis through B7‐H3 in clear cell renal cell carcinoma" was retracted in 2025. Reasons: duplicated images; unreliable data; unreliable results or conclusions.

## Discussion

Previous study reported that B7‐H3 is an important immune regulatory molecule. Initial studies have shown that B7‐H3 can selectively promote T cells to secrete IFN‐γ and can play an important role in the antitumor immune response [32, 33]. However, subsequent studies have found that knocking out the B7‐H3 molecule can aggravate the inflammatory response, and they confirm that this molecule is mainly involved Th2 subgroup differentiation [7, 34]. The main function of B7‐H3 is increasingly believed to inhibit T cell immune response, which is a cosuppressive molecule [35, 36].

In addition to immune regulation, clinical significance of B7‐H3 expression and its role in tumor biology have received increasing research attention. In related studies, B7‐H3 molecules are high expressed in tumor vasculature and metastatic lymph node tissues of ccRCC, colorectal cancer and pancreatic carcinoma [16, 37, 38]. B7‐H3 can promote tumor angiogenesis and reduce the sensitivity of metastatic tumors to therapeutic drugs, pointing to an adverse effect on the prognosis of patients, and is therefore an important indicator in predicting cancer progression [13, 39].

The expression of B7‐H3 in tumor vascular endothelium and its clinical significance are gradually becoming a new research hotspot. Seaman *et al*. [14] applied high‐throughput screening techniques to analyze differentially expressed molecules between colon cancer vascular endothelium and normal blood vessels; in this study, B7‐H3 has been identified as a membrane molecule with the most significant up‐regulation of expression. In addition, abnormally expressed B7‐H3 also has been detected in a variety of tumor vascular endothelial cells, which suggested that its expression is closely related to clinical prognosis. Chen *et al*. [41] and Kapoor *et al*. [40] showed that B7‐H3 can promote the adhesion, invasion and metastasis of tumor cell lines by adhering to the extracellular matrix [40, 41]. Previous studies demonstrated that, in prostate cancer, using small interfering RNA to silence B7‐H3 can reduce the adhesion of FN to PC‐3, indicating that B7‐H3 mediates the extracellular matrix FN to regulate cell adhesion during tumor metastasis [15].

Recently, it has been shown that B7‐H3 can maintain the continuous phosphorylation of STAT‐3 (Tyr705) and play a critical role in antagonizing the chemical drug docetaxel‐induced cell apoptosis [42]. Because the receptor or ligand to which the molecule directly binds has not been identified so far, the biological mechanism of how B7‐H3 exerts the earlier effects still remains unclear. Currently, although there is no unanimous conclusion on the regulation of B7‐H3, studies on the regulation of B7‐H3 by microRNAs have emerged. In 2009, Xu *et al*. [33] showed that miR‐29 can regulate the expression of B7‐H3 [43], and then Yang *et al*. [44] further found that miR‐199a regulates biological functions of cells through targeting B7‐H3. However, the expression of B7‐H3 was not regulated by microRNA only [44], as the concentration of cytokines around cells, stimulation of B7‐H3 on antibodies and the expression of intracellular proteins can all affect the expression of B7‐H3.

The article "Fibronectin enhances tumor metastasis through B7‐H3 in clear cell renal cell carcinoma" was retracted in 2025. Reasons: duplicated images; unreliable data; unreliable results or conclusions.

This study, for the first time, found that B7‐H3 bound to exogenous FN, and confirmed that kidney cancer cells with high expression of B7‐H3 adsorbed a higher level of extracellular matrix FN and significantly promoted the invasion and metastasis of ccRCC cells in a FN‐dependent manner. The most significant feature of this study was the discovery of a new mechanism for this molecule in promoting tumor invasion and metastasis.

We found earlier the use of anti‐FN polyclonal antibody as the coating antibody, that the exogenous B7‐H3 fusion protein (with IgG fusion protein as the isotype control) was added after BSA blocking, and that the HRP labeled anti‐B7‐H3 single detection analysis. It was found that both the control group and the B7‐H3 fusion protein group produced positive reactions. However, in the earlier experiment, using FN mAb instead of FN polyclonal antibody led to a positive reaction only in the B7‐H3 fusion protein group. Based on these findings, we speculated that FN and B7‐H3 protein may exist in the form of a natural complex. Through database analysis, we found that B7‐H3 and FN were significantly positively correlated in ccRCC, which may be explained by the coexpression between B7‐H3 and FN, or that B7‐H3 and FN were expressed in similar tumor subtypes and were regulated by similar mechanisms. To verify the earlier hypothesis, we performed the co‐IP experiment to validate the interaction of B7‐H3 and FN. However, the combination of FN and B7‐H3 did not necessarily produce a functional effect, and the combination of the two still requires further analysis.

Previous studies demonstrated that both B7‐H3 and FN promote tumor cell invasion and metastasis [25, 45, 46]. To investigate whether the functional interaction of B7‐H3 and FN could promote cell invasion, we constructed ccRCC cell lines differentially expressing B7‐H3, with exogenous FN for intervention. The data revealed that the high‐expressed B7‐H3 ccRCC cell line showed a significantly higher level of adsorbed FN than the low‐expressed B7‐H3 ccRCC cell group, proving their interaction at a cellular level. Further experiments confirmed that in the high‐expressed B7‐H3 group, more exogenous FN was deposited on the cell membrane surface. FN enhanced the migration and invasion of ccRCC cells and promoted the up‐regulation of PI3K/AKT and p38/ERK MAPK signaling pathways phosphorylated proteins. However, there was no obvious deposition of exogenous FN and biological changes in the low‐expression B7‐H3 group. Although this result may be because of the possibilities that ccRCC cells become another subtype of ccRCC tumor cells after knocking down the expression of B7‐H3, and this type of cell has a limited response to exogenous FN, which might lead to the binding of exogenous FN to the cells. Therefore, knocking down B7‐H3 may result in the decrease of FN deposition, which in turn reduced the phosphorylation of related signaling pathway proteins and inhibited the EMT process.

The article "Fibronectin enhances tumor metastasis through B7‐H3 in clear cell renal cell carcinoma" was retracted in 2025. Reasons: duplicated images; unreliable data; unreliable results or conclusions.

Our study explored the clinical significance and prognostic relationship of B7‐H3 in ccRCC and also was a novel discovery of interaction of B7‐H3 with plasma FN in promoting ccRCC metastasis. Cotargeting FN and B7‐H3 could contribute to new therapeutic intervention strategies for ccRCC treatment.

## Conflict of interest

The authors declare no conflict of interest.

## Author contributions

JX and MS conducted experiments and were responsible for data acquisition and manuscript writing. DZ was responsible for data interpretation and data analysis. CC and SL helped with statistical analysis. GZ conceived and designed the study and critically revised the manuscript for important intellectual content. All authors read and approved the final manuscript.

## Supporting information


**Fig**. **S1**. Lentiviral‐mediated RNAi efficiently suppresses B7‐H3 expression in the 786‐O and ACHN cell lines. (A,B) Gene knockdown verification at the mRNA level by RT‐qPCR analysis. Values are expressed as means ± SD (*t* tests, *n* = 3), **P < 0.01; ***P < 0.001 B7‐H3 control vs. B7‐H3‐KO group.
**Fig. S2**. Small interfering RNA silences the expression of FN. (A,B) Knockdown efficiencies of FN in 786‐O and ACHN cells assayed by western blotting. Values are expressed as means ± SD (*t* tests, *n* = 3), **P < 0.01; ***P < 0.001 FN control vs. si‐FN group.
**Table S1**. Primers for RT‐qPCR.

## Data Availability

The data that support the findings of this study are available on request from the corresponding author. The data are not publicly available because of privacy or ethical restrictions.
